The article "Detection Method of Athlete Joint Injury Based on Deep Learning Model" was published in 2022. Journal: Comput Math Methods Med.

# Detection Method of Athlete Joint Injury Based on Deep Learning Model

**DOI:** 10.1155/2022/8165580

**Published:** 2022-09-02

**Authors:** Jianjia Liu, Xin Yang, Tiannan Liao, Yong Huang

**Affiliations:** ^1^Department of Orthopedics, Hospital of Chengdu University of Traditional Chinese Medicine, Chengdu 610072, China; ^2^School of Public Affairs & Law, Southwest Jiaotong University, Chengdu, 610000, China

## Abstract

The research on accurate and intelligent segmentation of knee joint MRI images is of great significance to reduce the work intensity of clinical doctors and nurses. In order to solve the problem that knee joint MRI image segmentation model needs a large number of high-quality tagged images and excessive labeling workload, a semisupervised learning segmentation network model based on 3D scSE-UNet is proposed. The model adopts a self-training semisupervised learning framework and adds a cSE-block+ module on the basis of the 3D UNet model. This module can enhance the effective features of the feature image from two aspects of space and channel, while suppressing irrelevant features and preserving image edge information more completely. In order to solve the problem of rough edge of pseudolabel caused by model segmentation, a fully connected conditional random field is added to refine the edge of pseudolabel in the process of model training. The effectiveness of the model is verified by open source MRNet dataset and OAI dataset. The results show that the proposed model can achieve the segmentation effect of fully supervised learning through a small number of labeled images and effectively reduce the dependence of knee joint MRI image segmentation on expert labeling data.

## 1. Introduction

Knee joint is one of the most important composite joints in human body [1]. Most of the complex human movements are inseparable from the knee joint, and it is also the most important load-bearing joint [2]. For athletes who take various sports as their professions, the health of knee joints and the early detection and treatment of injuries are particularly important [3]. After knee joint injury caused by exercise, timely and accurate professional evaluation of anterior cruciate ligament injury is of great significance for medical staff to choose the best treatment and to prevent the impact of injury on athletes' career [4]. In medicine, the examination of knee joint injury and lesion usually depends on magnetic resonance imaging (MRI). The advantage of MRI over arthroscopy is that it can clearly display articular cartilage and bone areas [5]. Theoretically, the knee joint history of patients and the pathological changes occurred during the occurrence of knee joint abnormalities can play a very important role in the diagnosis of specific knee joint problems. However, in the actual operation, there is still a case of low diagnostic sensitivity. The doctor will inevitably touch the pain point of the patient's knee joint in the clinical examination, which will increase the pain of the patient. This problem hinders clinical examination [6].

The article "Detection Method of Athlete Joint Injury Based on Deep Learning Model" was published in 2022. Journal: Comput Math Methods Med.

Knee arthroscopy is one of the commonly used methods in the diagnosis of knee joint diseases. However, since the introduction of MRI technology, this relatively noninvasive diagnostic tool has gradually replaced invasive arthroscopy [7]. It visualizes the abnormal problems of the knee joint by presenting a high-resolution image of the interior of the knee joint. The application of MRI provides reference and guidance for orthopedic experts in the preliminary diagnosis, treatment, and prognosis of meniscus, ligament, and tendon-related problems. At the same time, the cost of MRI of the knee joint is also slowly falling. Coupled with its noninvasive advantages, the current medical diagnosis and treatment is not only in the preoperative MRI examination of patients but also began to be used as an auxiliary diagnosis in the preliminary diagnosis of knee joint diseases.

In recent years, deep learning methods have made great progress in the field of computer vision, such as object detection [8], human posture estimation [9], or semantic segmentation [10]. Similarly, in the field of medical images, deep learning has achieved excellent results in disease classification [11, 12], cancer detection [13, 14], organ segmentation [15], and image reconstruction [16]. The application of deep learning in knee joint MRI image analysis is becoming a hot research content. Li et al. [17] used the multimode feature fusion model in deep learning to diagnose the injury of knee joint MRI images. The results show that the prediction accuracy of the model in knee joint tear is 96.28%, and it is proved that the MRI image classification model based on depth learning can accurately classify the type of anterior cruciate ligament injury. Chaudhari et al. [18] compared deep learning super resolution (DLSR) with conventional knee MRI and found that conventional MRI was 92% accurate in evaluating knee cartilage, meniscus, bones, ligaments, extensors, and synovium, while DLSR was consistent with its accuracy. This shows that DLSR can simplify the diagnosis of knee joint MRI. Yang et al. [19] applied the conditioned adversarial network to 30 groups of clinical MRI images and successfully carried out automatic cartilage segmentation through model training. The results show that transfer learning can achieve the same segmentation accuracy as human when the number of samples is small. Iqbal et al. [20] aimed at automatically monitoring the health degree of human knee synovial fluid and adopted the transfer learning model to solve the problem that it is difficult to label data sets on a large scale in medical images. At the same time, it is also proved that the model has a good recognition of human knee joint synovial fluid.

The article "Detection Method of Athlete Joint Injury Based on Deep Learning Model" was published in 2022. Journal: Comput Math Methods Med.

The above research has made some progress in knee joint MRI image segmentation, but still does not solve a common problem. On the one hand, for MRI images, it is difficult for a medical institution or imaging center to have enough tagged and untagged data. However, the MRI images from different image centers will be affected by imaging equipment, imaging protocols, and operating technicians, which makes it difficult for the model to train well. The main reason for this effect is that the resolution of MRI image is different due to the difference of imaging equipment and imaging protocol. Different levels of operators easily lead to differences in the degree of presentation of lesions on MRI images. On the other hand, well-trained models should be more robust to adapt to different sources of data.

Based on the above problems, we use two open knee joint MRI data sets from different sources, namely, MRNet and OAI datasets for semisupervised learning. The main difference between the two datasets is that each sample is marked with an exception in the MRNet dataset, while the OAI dataset is untagged. In this paper, the semisupervised learning knee joint segmentation method of self-training 3D scSE-UNet segmentation network is used to train part of the MRI dataset as tagged data and the other part as untagged data. In the process of self-training, a fully connected conditional random field is added to refine the predicted pseudolabel edge to improve the accuracy. After training, the model can achieve the purpose of effectively training 3DscSE-UNet with a small amount of labeled data and a large number of unlabeled data, so as to improve the accuracy of knee joint segmentation (abnormalities, ACL tears, and meniscus tears) and reduce the dependence of deep learning image segmentation methods on label data.

## 2. Methods

### 2.1. Self-Training Semisupervised Learning Segmentation

Reasonable and effective use of the effective information in MRI images is helpful to improve the segmentation accuracy of the target region. Therefore, the self-training method is used to segment the image. Self-training is a representative method in semisupervised learning. It trains the untagged data through a small amount of tagged data to produce pseudotags. Combined with true tags to pseudotags, the segmentation model is trained. In the process of segmentation, a small amount of tagged data is input into the segmented network while a large amount of untagged data is input to carry out cyclic iterative training of the network.

The article "Detection Method of Athlete Joint Injury Based on Deep Learning Model" was published in 2022. Journal: Comput Math Methods Med.

In this study, the self-training semisupervised segmentation method is shown in Figure 1. In the figure, *X* represents the MRI image, and *Y* tags it. In self-training semisupervised learning, two datasets are used, which are shown in the following formula.

(1) $$\begin{array}{c} \text{Tagged data}:D_{L}=\left\{X_{L},Y_{L}\right\}, \end{array}$$

(2) $$\begin{array}{c} \text{Untagged dataset}:D_{U}=\left\{X_{U}\right\}. \end{array}$$

Among them, the label in the tagged data set comes from the expert, hereinafter, referred to as the truth label. The untagged dataset contains only grayscale images. The goal of this training is to predict the untagged data set and get pseudotags by training the 3D scSE-UNet model. Finally, the pseudotag is extended to the untagged dataset.

The specific training steps can be subdivided into 5 steps: (1) using tagged *D*_*L*_ of partial data in MRNet dataset to train 3D scSE-UNet model. (2) The untagged dataset is randomly divided into several subdatasets. Input the subdataset into the 3DscSE-UNet model for prediction, and the prediction result of the response can be obtained. It is important to note that the subdataset contains tagged data from MRNet and untagged dataset from OAI. (3) Inputing the segmentation result into dense CRF for edge refinement to make it closer to the true value label. Finally, the refined pseudotags are added to equation (3) to build a new dataset, namely, equation (4). (4) Adding equation (5) to *D*^*i*+1^_trian_ to build equation (6). Use *X* for the next round of training. (5) Inputing the updated training set into 3DscSE-UNet model for training again. After the training is completed, enter the next batch of untagged data and repeat the above steps until all untagged data produces false tags. In the process of training, because the pseudotag is extended to the training set, the model can continuously obtain new features and enhance the robustness of the model.

(3) $$\begin{array}{c} {D^{i}}_{U}=\left\{{X^{i}}_{U}\right\}, \end{array}$$

(4) $$\begin{array}{c} {D^{i}}_{U}=\left\{{X^{i}}_{U},{Y^{i}}_{U}\right\}, \end{array}$$

(5) $$\begin{array}{c} {D^{i}}_{U}=\left\{{X^{i}}_{U},{Y^{i}}_{U}\right\}, \end{array}$$

(6) $$\begin{array}{c} {D^{i+1}}_{trian}={D^{i}}_{trian}+{D^{i}}_{U}. \end{array}$$

In the formula, *i* represents the *i* iteration, *i* + 1 represents the *i* + 1 iteration, *U* represents unlabeled data, *D* represents the data set, and trian represents the training set.

The article "Detection Method of Athlete Joint Injury Based on Deep Learning Model" was published in 2022. Journal: Comput Math Methods Med.

#### 2.1.1. DscSE-UNet Segmentation Network

In the self-training learning segmentation method involved in this study, scSE-block+ is combined with 3D UNet. ScSE is an attention module which integrates channel dimension and spatial dimension. Its main function is to enhance the meaningful features and suppress the useless features, so as to improve the accuracy. The two constitutes the 3DscSE-UNET segmentation network model. The schematic diagram of its structure is shown in Figure 2. The structure design of the network model is similar to that of 3DUNet, which adopts U-shaped structure. In the figure, the arrows represent the connection mode of different processing layers and the input direction of the feature map. The text above the arrow represents the number of channels of the feature map.

The difference between the new model and the 3D UNet model structure is that a scSE-block+ is added at the end of each hop connection layer in the 3D UNet decoding part, that is, the red square in the figure. The processing layer resets the weight of the feature channel of the input image to strengthen the effective features while weakening the useless features, so as to improve the ability of self-training semi-supervised learning network to learn effective features and improve the accuracy.

The decoding layer of the model performs the operations of generating feature maps and extracting features from MRI images of the input model by up/downsampling techniques, respectively. Among them, four lower sampling layers are designed in the coding layer, and each lower sampling layer is composed of two convolution layers. The convolution layer is responsible for extracting different levels of image features and activating them through the ReLU function. After two convolution layers, a maximum pool layer with a step size of 2 is connected to compress the features and reduce the dimension. In the decoding layer, each layer consists of an upper sampling layer with a step size of 2 and 2 convolution layers with a step size of 3 × 3 × 3. After each convolutional layer, a ReLU function is set to activate it. Through the way of jump connection, the model combines the feature images obtained by the coding layer and the feature images obtained by the decoding layer with the same resolution. The combination of shallow and deep features to refine the image allows more texture information of the original image to spread in the high-resolution layer. Finally, the fused features are input into the scSE-block+ module to suppress the unimportant features and improve the accuracy of the segmentation results.

### 2.2. scSE-Block+ Module

In the proposed self-training semisupervised learning model, a total of 4 scSE-block+ modules are used, and their structure is shown in Figure 3. The main reason for setting up four scSE-block+ modules is that the module can perform its function better in front of the upper sampling layer. This module can calculate the feature space domain and feature channel domain at the same time. By learning the importance of each feature, the feature graph is recalibrated. ScSE-block+ is the weight of channel SE module and spatial SE module.

The article "Detection Method of Athlete Joint Injury Based on Deep Learning Model" was published in 2022. Journal: Comput Math Methods Med.

As can be seen in Figure 3, we have improved the cSE-block, that is, the part of the figure marked as a dotted line. On the basis of the original cSE-block module, the model adds a global maximum pool layer, which is marked as a red square in the figure. The newly added pooling layer is parallel to the original global average pooling layer of cSE-block. In the process of compressing spatial information, the selection of spatial feature tensor is different between the maximum pool layer (MPL) and the average pool layer (APL), which makes up for the problem that the original cSE-block module is not comprehensive.

The essence of MPL is to calculate the maximum value of the whole feature graph. Because the edge of the feature graph may produce the largest eigenvalue, MPL can retain the texture and edge features of the image to the maximum extent. The essence of APL is to calculate the average value of the whole feature graph and pay more attention to the downsampling of the whole feature. Therefore, APL can better retain the background of the feature map. MPL and APL are visible. In the task of extracting image edge information, MPL is more effective than APL. If the two are processed in parallel, the dual characteristics of edge and background can be retained. It plays a significant role in improving the performance of the model. Specifically, cSE-block evaluates the importance of channels by compressing spatial information. The module inputs the feature graph of *H* × *W* × *S* × *C* into a MPL and an APL in parallel. Among them, *H* × *W* × *S* × *C* represents the length, width, depth, and number of channels of the feature graph, respectively. MPL and APL compress the global spatial information in the lattice channel to a tensor value, respectively. The eigenvalue produced by this process is 1 × *C*. Then, these eigenvalues are convoluted in three dimensions. The convolution kernel size is 1 × 1 × 1 and the number of channels is *C*. Finally, the features obtained by convolution operation are activated by ReLU function, respectively. After the above convolution operation, two tensors of 1 × 1 × 1 × *C* with different values but with the same dimension are obtained. After the two tensors are added, the input sigmoid layer is normalized. By multiplying the normalized value with the original eigenmatrix, the unimportant information in the channel can be suppressed obviously, and the information in the important channel can be preserved losslessly. The important information mentioned here, in this study, refers to the information related to the purpose of model training.

The article "Detection Method of Athlete Joint Injury Based on Deep Learning Model" was published in 2022. Journal: Comput Math Methods Med.

In image segmentation, the spatial information of each pixel will provide more information. Therefore, the parallel sSE-block module is introduced into the research. This module can evaluate the importance of spatial location by compressing channel information. For the feature map of an input module, the module realizes space extrusion through convolution operation. Then, it is normalized by sigmoid. Finally, it is multiplied by the original characteristic tensor.

### 2.3. Fully Connected Conditional Random Field

In the self-training model, the unlabeled samples segmented by the algorithm are prone to missegmentation. After the missegmented samples are generated, they will still be extended to the training set to participate in the new round of training as the mark of the next round of samples. This causes the model to learn the wrong labels and make the errors accumulate, even magnify the errors.

In order to solve the above problems, it is necessary to improve the accuracy of pseudotags to the maximum extent. The fully connected conditional random field can optimize the rough and uncertain tags in the pseudotags, correct the missegmented regions, improve the positioning characteristics of the network, and then get more accurate and detailed pseudotags. In this study, we introduce fully connected conditional random field (dense CRF) in the self-training process to refine the pseudotags obtained in each iteration of the self-training process.

The core of dense CRF algorithm is to calculate the relationship between pixels and pixels. The two pixels with high degree of similarity are assigned the same label, and the probability of being segmented is low. However, when different labels are assigned between the two pixels with lower similarity, the probability of being segmented increases. The energy function of dense CRF algorithm is shown in the following formula:

(7) $$\begin{array}{c} E\left(x\right)=\underset{i}{\sum }\psi_{\text{u}}\left(f_{i}\right)+\underset{i<j}{\sum }\psi_{\text{p}}\left(f_{i},f_{j}\right), \end{array}$$

(8) $$\begin{array}{c} \psi_{\text{u}}\left(f_{i}\right)=-\log P\left(f_{i}\right). \end{array}$$

*ψ*_u_(*f*_*i*_) represents the unary potential energy, and it is mainly used to calculate the classification probability of pixel points, as shown in equation (8), and *f*_*i*_ represents the prediction result of pixel *i* by the segmentation model. *P*(*f*_*i*_) represents the probability that the predicted result of pixel *i* is *f*. *ψ*_p_(*f*_*i*_, *f*_*j*_) represents the binary potential energy between pixel *i* and the predicted result *f*_*i*_, *f*_*j*_ on pixel *j*, which can describe the relationship between the two pixels

(9) $$\begin{array}{c} \psi_{\text{p}}\left(f_{i},f_{j}\right)=\mu \left(f_{i},f_{j}\right)\left[\begin{array}{c} \omega_{1}\exp\left(-\frac{{\left\|x_{i}-x_{j}\right\|}^{2}}{2\sigma_{\alpha }^{2}}-\frac{{\left\|y_{i}-y_{j}\right\|}^{2}}{2\sigma_{\beta }^{2}}\right)+\\ \omega_{2}\exp\left(-\frac{{\left\|x_{i}-x_{j}\right\|}^{2}}{2\sigma_{\gamma }^{2}}\right) \end{array}\right]. \end{array}$$

In the formula, *ω*_1_ and *ω*_2_ are linear combination weights; *μ* is the label compatibility function, and *μ*(*f*_*i*_, *f*_*j*_) is the label compatibility item, which restricts the condition of conduction between pixels, when *f*_*i*_ ≠ *f*; it has the value 0; the proximity and similarity between pixels are controlled by coefficients *σ*_*q*_ and *σ*_*g*_; *σ*_*γ*_ = 1, which can remove small independent regions. *X*_*i*_ and *X*_*j*_ are the position information of pixel *i* and pixel *j*, respectively, and *y*_*i*_ and *y*_*j*_ are the intensity values of pixel *i* and pixel *j*, respectively. The binary potential energy function will pay more attention to the pixels with similar position *x* and similar intensity *y* but with different marks *f*. The smaller the energy *E*(*x*) is, the more accurate the predicted category label *x* is.

The article "Detection Method of Athlete Joint Injury Based on Deep Learning Model" was published in 2022. Journal: Comput Math Methods Med.

In the process of segmenting MRI image by dense CRF module, the unary potential can represent the probability distribution map. Specifically, it is the result obtained by the input softmax function of the characteristic graph output of the model. The position information and gray information extracted from the original image are assigned to the binary potential energy. With the combination of unitary potential energy and binary potential energy, the relationship between pixels can be comprehensively evaluated, and the results can be optimized. In this study, the model uses the iterative energy function *E*(*x*) to find the minimum solution of each image through five iterations to identify the most likely category of each pixel in the MRI image. Finally, each optimized prediction result is added to the self-training learning as a pseudotag.

## 3. Model Training and Evaluation Method

### 3.1. Model Training Parameter Setting

In the aspect of model parameter setting, the unlabeled data set is divided into 5 subdata sets. Each data set is input into the model in turn for prediction, and the corresponding prediction results (segmentation results) are produced. In the process of training, the gradient descent algorithm built into Adam optimizer is used to find the minimum value of network parameter error function. Set the network learning rate of the model to 0.0001 epoch; set the training number (epoch) to 150; set the batchsize to 1; and stop training after reaching the maximum number of cycles. The setting of training cycle, training times, and batch size is mainly based on the experience of previous studies. All data set processing, model training, verification, and evaluation are done on the same computer.

The article "Detection Method of Athlete Joint Injury Based on Deep Learning Model" was published in 2022. Journal: Comput Math Methods Med.

### 3.2. Evaluation Index

The quantitative indexes for evaluating the semisupervised 3DscSE-UNet model are average symmetrical surface distance (ASSD), 95 percentile Hausdorff distance (HD95), and disc coefficient (DC), respectively. ASSD is used to calculate the average surface difference between segments. Hausdorff distance calculates the maximum point distance between segments. DC focuses on evaluating the degree of overlap between the two groups of segmentation results. Therefore, these three indicators are complementary and trinity.

ASSD calculates the overall average of the distance from *∂G* to the point on *∂S* and the distance from the boundary of *S*(*∂S*) to the point on *G*(*∂G*) boundary, as shown in the following formulas:

(10) $$\begin{array}{c} \text{ASSD}\left(G,S\right)=\frac{\sum_{g\in \partial G}\underset{s\in \partial S}{\min}\left\|s-g\right\|+\sum_{s\in \partial S}\underset{g\in \partial G}{\min}\left\|g-s\right\|}{\left|\partial G\right|+\left|\partial S\right|}, \end{array}$$

(11) $$\begin{array}{c} \left\|\overset{⟶}{a}\right\|=\sqrt{\overset{n}{\underset{i}{\sum }}{\left(a_{i}\right)}^{2}}=\sqrt{{\left(a_{1}\right)}^{2}+{\left(a_{2}\right)}^{2}+\cdots +{\left(a_{n}\right)}^{2}}. \end{array}$$

In the formulas, *G* is the segment of basic facts, and *S* is the segment to be predicted. |·| represents the cardinality of the set. The smaller the calculation result of ASSD is, the better the split boundaries are consistent with each other.

The Hausdorff distance is calculated by the following formula:

(12) $$\begin{array}{c} \text{HD}\left(G,S\right)=\max\left(h\left(G,S\right),h\left(S,G\right)\right). \end{array}$$

Among them, the calculation method of *h*(*G*, *S*) is

(13) $$\begin{array}{c} h\left(G,S\right)=\underset{g\in G}{\max}\underset{s\in S}{\min}\left\|g-s\right\|. \end{array}$$

HD is the module for calculating the maximum segmentation error. Because HD is highly sensitive to outliers, and outliers in HD are replaced with 95% of the maximum in HD95.

The article "Detection Method of Athlete Joint Injury Based on Deep Learning Model" was published in 2022. Journal: Comput Math Methods Med.

The calculation model of DC is

(14) $$\begin{array}{c} \text{DC}=\frac{2\left|G\cap S\right|}{\left|G\right|+\left|S\right|}. \end{array}$$

DC is a widely recognized index in the research of knee joint MRI image segmentation. Its scope is [0,1], where 0 means undivided, and 1 indicates that the segmentation is completely consistent.

## 4. Results and Analysis

### 4.1. Results

In order to avoid the chance of the training results of the model, five experiments were carried out based on the model proposed in the study, and the average value of the five experiments was taken as the result. The model involved in this study is trained on NVIDIA RTX3090 GPU, and the training time of one model is about 26 hours. Once the model is trained, the average segmentation time of each test image is less than 2 s.

In each experiment, 20 images from the tagged MRNet dataset and 26 images from the OAI dataset were randomly selected as the test set. The number of randomly selected images from both datasets is 1/5 of the labeled images in the dataset. 100 images were selected from MRNet data set, and 50, 40, 30, 20, and 10 MRI images and their truth tags were randomly selected as tagged data. The remaining 50, 60, 70, 80, and 90 MRI images were used as untagged data to form five training sets with different proportion of tagged data. The model obtained under five kinds of training conditions was used to predict the test set, and the segmentation results were compared with those obtained by 3D UNet fully supervised learning. Full-supervised and semisupervised methods show different performance in knee joint MRI image segmentation, as shown in Figure 4.

As can be seen from Figure 4, when the proportion of label data in knee joint segmentation reaches 30%, ASSD = 2.431, HD95 = 1.596 mm, and DC = 0.941. The prediction result of full supervision method is ASSD = 1.974, HD95 = 2.697 mm, and DC = 0.950. It can be seen that when the labeled data accounts for 30% of the training set, the evaluation index of semisupervised learning segmentation result is better than that of fully supervised learning method.

In order to compare the segmentation performance of the model under different percentages of labeled data in the training set, based on the study of the proposed model, the DC values under different conditions are obtained through training, and the DC changes under different ratios are drawn, as shown in Figure 5. As can be seen in the figure, the DC value increases with the increase of the proportion, and the growth rate decreases gradually. When the proportion is less than 40%, the DC value increases with the increase of the proportion, and the rising speed increases from 0.902 to 0.946. When the proportion is more than 40%, the growth rate slows down. Until the proportion reaches 100%, the fully supervised model DC = 0.950.

The article "Detection Method of Athlete Joint Injury Based on Deep Learning Model" was published in 2022. Journal: Comput Math Methods Med.

### 4.2. Performance Comparison between Semisupervised Learning and Fully Supervised Learning

Comparing the performance of the self-training semisupervised model with the full-supervised model, we can better verify the effectiveness of the self-trained semisupervised model. For this reason, the 3D scSE-UNet segmentation network model is used to train the semisupervised model and the full-supervised model, respectively, and the performance of the semisupervised model and the full-supervised model is compared. The comparison results are shown in Figure 6.

As can be seen in the figure, when the network model is segmented by 3DscSE-UNet at the same time, and the label data are the same, the performance of the semisupervised learning model is better than the fully supervised learning model. The main reason is that the semisupervised learning model can improve the segmentation performance through the effective use of unlabeled data, especially in the case of less tagged data. In the case of more tagged data, the segmentation accuracy of semisupervised learning model is not significantly higher than that of fully supervised learning, especially when the proportion of tagged data is 50%. The main reason for this phenomenon is that when there are a lot of labeled data, the fully supervised learning model can segment the image more accurately through training, and there is little room for semisupervised learning to improve.

### 4.3. Comparison of Segmented Networks with scSE-Block+

In order to understand the improvement effect of the scSE-block+ module added in this study on the self-training semisupervised learning network model, the model is used to compare the segmentation ability of the model before and after adding. The training adds 30% of the training set with tagged data, and the result is shown in Figure 7. As can be seen in the figure, the ASSD value, HD95 value, and DC value of the model are significantly improved after the addition of scSE-block+ module. It can be seen that the scSE-block+ module can make more full use of the channel and spatial information in the feature graph.

Because the global maximum pool layer is added to the scSE-block module in the study, it is necessary to verify and compare the performance of the module before and after the addition and evaluate the impact of the improved module on the segmentation results. This verification uses a training set with a 30% proportion of labeled data, and the verification result is shown in Figure 8. As can be seen in the figure, the effect of image segmentation is better after adding the global maximum pool layer. In the process of feature extraction, using the global maximum pool layer can retain more abundant edge information and optimize the segmentation effect of the segmentation model on the target region.

The article "Detection Method of Athlete Joint Injury Based on Deep Learning Model" was published in 2022. Journal: Comput Math Methods Med.

### 4.4. Dense CRF Performance Comparison

In order to refine the segmentation results of pseudo tags, a dense CRF module is added to the research model. In order to analyze the thinning effect of pseudotags, the segmentation effects of pseudotags before and after thinning are compared, as shown in Figure 9. The training set used in the comparative study is 30% of the labeled data.

As can be seen in the figure, the performance index of the segmentation result optimized by dense CRF module has been improved compared with that before optimization. From the point of view of the segmentation results, the optimized segmentation results are closer to the truth label at the edge and even overlap with the truth label. For the part of the segmentation result with poor edge, the dense CRF module can modify it to make it closer to the truth label.

By calculating the relationship between a single pixel and all other pixels, the dense CRF module establishes a dependency on all pixel pairs in the image and then finely processes the probability map of the segmentation network prediction. Although the overall segmentation accuracy is not greatly improved by adding dense CRF module to the self-training semisupervised learning model, the edge thinning effect of the segmentation result is better.

### 4.5. Comparison of Time Performance of Models

In this study, the average image processing time of the four models involved in the study was compared. The four models are fully supervised 3DUNet model, semisupervised 3DUNet model, fully supervised 3DscSE-UNet model, and semisupervised 3DscSE-UNet model. One hundred untagged MRI images were randomly selected from OAI datasets to test the average processing time of the four models, and the results are shown in Figure 10. As can be seen from the figure, due to the addition of the scSE-block+ module, the average processing time of the 3DscSE-UNet segmentation model is longer than that of the 3DUNet model, but there is little difference between the two models, which is only 150 ms. Under the same segmentation model, the effect of semisupervised learning or fully supervised learning on the average image processing time can be ignored.

The improved training model can segment MRI images more accurately and can basically achieve automatic segmentation of MRI images. This study has some significance to reduce the workload of medical workers and reduce the misdiagnosis of knee lesions.

The article "Detection Method of Athlete Joint Injury Based on Deep Learning Model" was published in 2022. Journal: Comput Math Methods Med.

## 5. Conclusion

In order to solve the problem that MRI image segmentation needs large labeling data and time-consuming experts in the field of knee joint depth learning, this study proposes a semisupervised learning segmentation model of 3DscSE-UNet knee joint MRI image based on scSE-block+, which reduces the dependence on labeled data in knee joint depth learning research and draws the following conclusions.

The fully connected conditional random field improves the detail processing ability of the semisupervised 3DscSE-UNet model and improves the accuracy of generating pseudotags in the segmented network. The addition of pseudotags to the semisupervised learning model significantly improves the segmentation performance of the model and achieves the purpose of making a large number of predictions from a small amount of label data. Through the verification of the model, it is found that the segmentation effect of the model is similar to that of the fully supervised learning model in the case of learning a small amount of labeled data

By learning the relationship between different features, the semisupervised 3DscSE-UNet model can enhance the useful features while suppressing the irrelevant features and improve the accuracy of knee joint MRI image segmentation. The addition of scSE-block+ module in the semisupervised 3D scSE-UNet model increases the average image processing time of the model. No matter which supervision method is adopted, the image processing time of the 3D scSE-UNet model is 17.94% higher than that of the 3DUNet model, with a difference of 150 ms. However, under the same supervision mode, the segmentation performance of 3D scSE-UNet model is significantly better than that of 3D UNet model

The main disadvantage of the self-training semisupervised learning model is that if the unlabeled data is mistakenly segmented in the initial segmentation, the problem will be magnified in the subsequent model training process. The main reason for the amplification is that the initial error marker has the potential to act as a trusted label, allowing subsequent errors to accumulate. In this study, the dense CRF module is used to alleviate the problem. In the follow-up study, we will work to improve this problem.

## Figures and Tables

**Figure 1:** Training method of 3D scSE-UNet network model.

**Figure 2:** Outline of the structure of 3D scSE-UNet network model.

**Figure 3:** Schematic diagram of scSE-block+ structure of additional processing layer.

**Figure 4:** Performance comparison of prediction results of training sets with different ratios of labeled data (full 3D UNet refers to fully supervised 3D UNet model, full 3D scSE-UNet refers to fully supervised 3D scSE-UNet model, LP50 refers to semisupervised 3D scSE-UNet model and training set with 50% of tagged data, and the following labels are synonymous).

The article "Detection Method of Athlete Joint Injury Based on Deep Learning Model" was published in 2022. Journal: Comput Math Methods Med.

**Figure 5:** Dice score curve of 3D scSE-UNet with different proportions of labels.

**Figure 6:** Performance comparison of fully supervised and semisupervised segmentation under different label ratios (L10 reference training set uses only 10 cases of tagged data, no untagged data, and the following labels are synonymous).

**Figure 7:** Performance comparison of 3D UNet and 3D scSE-UNet segmentation results.

**Figure 8:** Comparison of segmentation results between scSE-block and scSE-block+.

**Figure 9:** Performance comparison of segmentation results between using and unusing dense CRF.

**Figure 10:** Average image processing time of different models.

## Data Availability

The experimental data used to support the findings of this study are available from the corresponding author upon request.
